# Predictive Model of Cerebral Vasospasm in Subarachnoid Hemorrhage Based on Regression Equation

**DOI:** 10.1155/2022/3397967

**Published:** 2022-04-26

**Authors:** Jianzhong Li, Kaiguo Zhou, Lei Wang, Qiumei Cao

**Affiliations:** Department of Emergency, Beijing Tongren Hospital, Capital Medical University, 100176, China

## Abstract

In order to explore the regression equation for the prediction model of subarachnoid hemorrhage and cerebral vasospasm, the nomogram prediction model of SCVS occurrence was established. This study is a retrospective analysis of 125 cases of aSAH admitted to a hospital; the patients were divided into SCVS group and non-SCVS group. Select SIRI as a simple and reliable marker of inflammation, analyze its correlation with SCVS and its predictive value, and analyze the predictive value of SIRI to SCVS through ROC curve. Based on the SIRI inflammation level and other related risk factors, a nomogram prediction model for the occurrence of SCVS was built. The experimental results show that the SIRI level of patients in the SCVS group was significantly higher than that of the non-SCVS group, and logistic regression analysis found that SIRI is an independent risk factor for SCVS. *SIRI* = 3.63 × 10^9^/*L* is the best cutoff value for diagnosing the occurrence of SCVS. When TC = 2.24 mmol/L and SIRI = 3.63 × 10%/L, its Youden Index is the largest (0.312, 0.296) and is the best cutoff value for predicting the occurrence of SCVS; at the same time, its prediction accuracy (area under the ROC curve (AUC)), sensitivity, specificity, the positive predictive value, and negative predictive value are 0.743, 72.70%, 80.10%, 77.53%, and 94.24% and 0.725, 70.60%, 76.90%, 73.49%, and 93.59%. Nomogram prediction model establishment and evaluation combined with the results of multifactor analysis are used to build an individual nomogram prediction model. The model has good prediction consistency (C-index = 0.685, *P* < 0.01). ROC analysis results showed that the model that combined SIRI and other standard variables (AUC = 0.896, 95% CI was 0.803-0.929, *P* < 0.001) was better than the model that did not combine SIRI (AUC = 0.859, 95% CI was 0.759-0.912, *P* < 0.001) and the model based only on SIRI (AUC = 0.725, 95% CI was 0.586-0.793, *P* = 0.001) has better predictive value for SCVS. Joint SIRI will optimize the prediction performance of the nomogram model and improve the early recognition and screening capabilities of SCVS.

## 1. Introduction

Subarachnoid hemorrhage (SAH) is one of the diseases that seriously endangers human life and health. According to statistics, about 50~70% of SAH patients have cerebral vasospasm (CVS) complications, and about 19~46% of SAH patients progressed to delayed ischemic neurological deficit (DIND) seriously affect the prognosis of SAH [1]. Animal experiments and clinical studies have found that the incidence of CVS is biphasic, with two peak periods of early onset and late onset. A few minutes to a few hours after SAH is the first high-incidence period, mostly in the blood vessels surrounding the ruptured aneurysm with the significance of the location of the tumor-bearing artery. The second high-incidence period is usually 4-16 days after SAH, with 7-10 days being the most common; most of them are diffuse and multisegmental and have no positioning value for the tumor-bearing artery [2]. According to Poiseuille's law of hemodynamics, the blood flow per unit time is proportional to the 4th power of the vessel radius. When the blood vessel diameter changes slightly, it can produce obvious changes in cerebral blood flow [3]. In CVS patients, vasospasm, narrowing of the tube diameter, will produce symptoms of insufficient blood supply to the brain, such as increased consciousness disturbance, cerebral edema, and cerebral infarction. It is still a challenge to diagnose CVS in a timely and accurate manner. Transcranial Doppler (transcranial Doppler sonography, TCD) and angiography (digital subtraction angiography, DSA) are currently recognized diagnostic methods, but there are still 1/4 to 1/3 of patients who cannot be diagnosed correctly; clinically, the diagnosis is often only after the deterioration of neurological function occurs; this has brought great passivity to the prevention and treatment. Therefore [4], it is very important to actively search for the risk factors of CVS and predict the occurrence of CVS. There are many risk factors for CVS that have been reported, including high blood pressure, diabetes, drinking, smoking, Hunt-Hess score, Fisher classification, fever, surgery, the total number of white blood cells, the total number of platelets, the location of the aneurysm, number of ruptures, and intraventricular hemorrhage; however, intracranial angiography is invasive and brings some risks [5]. The traditional clinical diagnosis method is based on the patient's clinical manifestations, the degree of SAH, the time after bleeding, and estimation of the weight of these objective factors such as TCD flow rate and Lindegaard rate [6]; and there are many studies focused on analyzing the relationship between TCD flow rate and CVS; however, these studies believe that only a very low or very high TCD flow rate can reliably predict CVS and did not fully consider the Lindegaard rate and VI; as a result, the diagnostic accuracy of CVS is not high. These studies also have limitations in statistical methods [7], most of the designs are retrospective studies, the appropriate statistical method should be a prospective cohort study, and a meaningful method has been used to integrate these factors and to meet the needs of clinicians to evaluate the risk of CVS in patients [8]. For more than 20 years, with the development of imaging technology, the performance of CT has improved a lot. In the current high resolution situation, grade 1 (no bleeding is seen) and grade 2 (bleeding thickness less than 1 mm) in the Fisher classification are rarely seen, and it is not exact to distinguish between grade 2 and grade 3 only by the thickness of the blood clot in the subarachnoid space [9]. Fisher classification has been unable to keep up with the needs of imaging progress. Especially when combined with intraventricular hemorrhage, the probability of concurrent CVS is high, and the Fisher classification cannot be well quantified. In 2001, Liang et al. revised the original Fisher classification, which is called the modified Fisher classification [10]. The modified Fisher classification is based on the thickness of blood in the subarachnoid space. As an independent risk factor for SCVS, the reason is presumed as follows: first, when the subarachnoid hemorrhage occurs, red blood cells are destroyed, producing a large amount of vasoconstrictors (oxyhemoglobin, adrenaline, norepinephrine, endothelin, etc.) to stimulate blood vessels, which causes strong and long-lasting spasms of blood vessels; secondly, the blood vessels running in the subarachnoid space, soaking in blood for a long time, can cause blood vessels to spasm. Furthermore, the blood clot in the subarachnoid space mechanically stretches and compresses the blood vessel wall, through nerve reflexes, etc. It can also cause vasospasm. Prolonged spasm further damages vascular endothelial cells, releasing more vasoconstrictors and creating a vicious circle and eventually SCVS. Many animal experiments and clinical studies have confirmed that the thickness and distribution range of hemorrhage determine the severity and range of vasospasm involvement to a certain extent; therefore, the modified Fisher classification, which is closely related to hemorrhage, can provide a good early warning of the occurrence of SCVS. Hunter-Hess classification is a commonly used indicator to reflect the severity of SAH patients [11]. Ryu et al. found that Hunter-Hess II~V level is an independent risk factor for SCVS [12]. According to Hsu et al., a multivariate analysis of 112 SAH patients found that Hunt-Hess IV-V grade and aging are independent risk factors for complication-like stroke [13]. The possible explanation is that there are many factors that affect Hunter-Hess classification, such as rebleeding, acute hydrocephalus, intracranial hypertension, fever, and electrolyte imbalance. Many factors can lead to a higher Hunter-Hess score; therefore, different statistical samples may draw different conclusions [14]. It shows that using Hunter-Hess classification to predict SCVS is less reliable. In addition to history of hypertension and location of aneurysm, there are differences between the two groups in 4-factor single factor analysis such as fever and ventricular hemorrhage; in the end, it failed to enter the multiple regression equation. The possible explanation is that their independent prediction of SCVS is still insufficient, not as sensitive as age and modified Fisher classification [15]. At the same time, it is not ruled out that some factors may be related to age and modified Fisher classification. Age and modified Fisher classification enter the equation; to a certain extent, it already contains information about the other 5 factors; this is exactly the advantage of using logistic regression. SCVS after subarachnoid hemorrhage is the result of multiple factors. Due to sampling errors, limited number of cases, etc., some possible risk factors have not been introduced. Therefore, to establish an accurate prediction model, it is still necessary to increase the sample size and continuously carry out prospective clinical verification. For patients with the above-mentioned risk factors in clinical work, the doctor should consider the poor clinical outcome. Diabetes in patients is due to relative or absolute lack of insulin, the organization's ability to use glucose decreases, lipoprotein lipase activity decreases, and elevated blood sugar and triglycerides gradually appear in vascular disease characterized by large and medium atherosclerosis, vascular endothelial dysfunction, and poor elasticity. The self-regulation function is impaired, resulting in ischemic or hemorrhagic cerebrovascular disease. At present, there is little literature on the relationship between diabetes history and CVS, and there is no conclusive conclusion. Most researches are on the relationship between blood glucose changes and CVS after SAH. It is generally believed that high blood sugar when SAH patients are admitted to the hospital is the result of a significant increase in catecholamines in the body and is a sign of SAH's serious condition, not a predictor of CVS. Based on the current research, in order to explore the regression equation for the prediction model of subarachnoid hemorrhage and cerebral vasospasm, the nomogram prediction model of SCVS occurrence was established. This study is a retrospective analysis of 125 cases of aSAH admitted to a hospital; the patients were divided into SCVS group and non-SCVS group. Select SIRI as a simple and reliable marker of inflammation, analyze its correlation with SCVS and its predictive value, and analyze the predictive value of SIRI to SCVS through ROC curve. Based on the SIRI inflammation level and other related risk factors, a nomogram prediction model for the occurrence of SCVS was built. There are 19 cases of aSAH patients complicated with SCVS after operation; the incidence rate was 15.20% (19/125). In SCVS group and non-SCVS group, smoking, hypertension, Hunt-Hess classification at the hospital, and the number of aneurysms, combined with intraventricular hemorrhage (IVH), have significant differences in modified Fisher classification, triglyceride (TC), monocyte count, and SIRI level (*P* < 0.01). Multivariate logistic regression analysis shows that, complicated with hypertension, Hunt-Hess classification in hospital (level IV~V), combined IVH, modified Fisher classification (IV~V grade), and high TG level and SIRI level are independent risk factors for SCVS in aSAH patients (*P* < 0.05). It has been verified that the model has good prediction consistency (C-index = 0.685, *P* < 0.01). ROC analysis results show that the model that combines SIRI and other standard variables (AUC = 0.896, 95% CI is 0.803-0.929, *P* < 0.001) is better than the model that does not incorporate SIRI (AUC = 0.859, 95% CI is 0.759-0.912, *P* < 0.001) and the model based only on SIRI (AUC = 0.725, 95% CI is 0.586-0.793, *P* = 0.001) has better predictive value for SCVS. Further conduct AUC hypothesis test, and it was found that the difference between AUC combined with/not combined with SRI model and AUC Yige with SIRI model was statistically significant (*Z* = 4.029, *P* < 0.001; *Z* = 3.734, *P* = 0.003). SIRI is closely related to SCVS after aSAH, and combined with SIRI, a Nomogram model will optimize the prediction performance and improve the early recognition and screening ability of SCVS occurrence.

## 2. Method

### 2.1. Information

Retrospectively analyze the data of 125 aSAH cases admitted to a hospital; among them, there were 45 males and 80 females, aged 24-86 years old, with an average of 56.0012.00 years old. Admission criteria are as follows: admitted to the hospital within 24 hours of onset and patients who were diagnosed with aSAH after admission and underwent early surgery within 3 days. Exclusion criteria are as follows: accompanied by serious medical diseases or other central nervous system diseases and before the operation, there was cerebral vasospasm. For those who died during hospitalization or withdrew from the study, the basic information is shown in Table 1.

### 2.2. Method

The patients were divided into SCVS group and non-SCVS group. Collect the age, gender, and personal history of the 2 groups of patients (smoking: in the past year, smoking ≥1 cigarettes a day on average; drinking: drinking ≥1 times a day on average), comorbidities (hypertension and diabetes), body mass index, Hunt-Hess classification at admission, aneurysm parameters (aneurysm diameter, location, and number), timing of surgery (ultraearly stage: <24 h; early stage: >24-72 h), surgical methods (craniotomy, clipping, and vascular embolization), and other information. Based on the characteristics of the first CT, the patients were modified Fisher grading, and record the presence or absence of intraventricular hemorrhage (IVH). At the same time, all patients collected 6 mL of venous blood after hospitalization for related laboratory tests, record in detail the blood sample test time, triglyceride (TC) level, white blood cell count, neutrophil count, lymphocyte count and monocyte count, and other laboratory indicators, and calculate SIRI: SIRI = Monocyte count × neutrophil count/lymphocyte count.

### 2.3. Statistical Methods

Use SPSS23.0 for data analysis. First, perform a normality test on all measurement data, the measurement data conforming to the normal distribution are expressed by the mean and standard deviation, and the comparison between groups is by *t* test [16]. Measurement data that does not conform to the normal distribution are represented by [*M*(*Q*_25_, *Q*_75_)]; the Mann-Whitney *U* nonparametric test was used for comparison. The counting data is represented by (*n*(%)); the *x*-test is used for comparison. The variables of *P* < 0.01 are included in the multivariate logistic regression analysis, and determine the risk factors for SCVS. According to the results of multifactor analysis, the rms installation package in R3.4.0 software was used to establish the nomogram prediction model. Finally, draw the receiver operating characteristic (ROC) curve to evaluate the predictive value of SIRI and predictive models for the occurrence of SCVS with inspection level *a* = 0.05, two-sided inspection.

## 3. Results and Analysis

### 3.1. Comparison of Basic Data of the Two Groups of Patients

There are 19 cases of aSAH patients complicated with SCVS after operation, the incidence rate was 15.20% (19/125) with Hunt-Hess grade, number of aneurysms, combined IVH, modified Fisher grade, TG, and monocyte count at admission of SCVS group and non-SCVS group, and there is a significant difference in SIRI level (*P* < 0.01) (see Table 2).

### 3.2. Multifactor Analysis

Multivariate logistic regression analysis shows that, combined with hypertension, Hunt-Hess classification in hospital (level IV-V), combined with IVH, modified Fisher classification (Level IV-V), and high TG level and SIRI level are independent risk factors for SCVS in aSAH patients (*P* < 0.05) (see Table 3).

### 3.3. ROC Cutoff Value

Plot the ROC curve to determine the index cutoff value, convert continuous variables (TG, SIRI) into binary variables. The results show that when TC = 2.24 mmol/L and SIRI = 3.63 × 10%/L, its Youden Index is the largest (0.312, 0.296) and is the best cutoff value for predicting the occurrence of SCVS; at the same time, its prediction accuracy (area under the ROC curve (AUC)), sensitivity, specificity, positive predictive value, and negative predictive value are 0.743, 72.70%, 80.10%, 77.53%, and 94.24% and 0.725, 70.60%, 76.90%, 73.49%, and 93.59%. Nomogram prediction model establishment and evaluation combined with multifactor analysis results are used to build an individual nomogram prediction model [17]. It has been verified that the model has good prediction consistency (C-index = 0.685, *P* < 0.01). ROC analysis results show that the model that combines SIRI and other standard variables (AUC = 0.896, 95% CI is 0.803-0.929, *P* < 0.001) is better than the model without SIRI (AUC = 0.859, 95% CI is 0.759-0.912, *P* < 0.001) and only the model based on SIRI (AUC = 0.725, 95% CI is 0.586-0.793, *P* = 0.001) has better predictive value for SCVS [18] (see Figure 1). A further hypothesis test of AUC was performed, and it was found that the difference between the AUC combined with/not combined with SIRI model and the AUC model based on SIRI only was statistically significant (*Z* = 4.029, *P* < 0.001; *Z* = 3.734, *P* = 0.003); however, there was no statistically significant difference between AUC combined with SIRI model and AUC without SIRI model (*Z* = 1.629, *P* = 0.1033).

During the occurrence and development of SCVS, neuroinflammatory response is the first important driving force. Therefore, by examining various inflammation indicators and their dynamic changes, it is of great significance to understand the patient's condition and predict the occurrence of SCVS [19]. With the deepening of research, the key roles of nuclear transcription factors and interleukins have gradually been emphasized. However, these testing items require special instruments and equipment, and the price is relatively high, and the clinical application is restricted. SIRI is a new type of complex inflammation marker based on traditional inflammatory cell count, which can more comprehensively reflect the body's inflammatory state. At the same time, it has the advantages of convenient detection, strong repeatability, and low price; it has become a good factor for predicting the occurrence, development, and prognosis of various diseases. In this study, SIRI was selected as a simple and reliable marker of inflammation, its correlation with SCVS and its predictive value have been analyzed, the results showed that the SIRI level of patients in the SCVS group was significantly higher than that of the non-SCVS group, and logistic regression analysis found that SIRI is an independent risk factor for SCVS. SIRI is a comprehensive index based on the absolute value of peripheral blood neutrophils, monocytes, and lymphocytes, representing different inflammatory and immune pathways in the body. The high SIRI state reflects the strong monocyte and neutrophil-mediated proinflammatory response and the weak or suppressed lymphocyte-mediated anti-inflammatory response; this aggravated the pathological degree of cerebral blood vessels after aSAH and induced the occurrence of SCVS. This study also analyzed the predictive value of SIRI to SCVS through the ROC curve. The results show that *SIRI* = 3.63 × 10^9^/*L* is the best cutoff value for diagnosing the occurrence of SCVS. When *SIRI* > 3.63 × 10^9^/*L*, it can be considered that the patient has a high inflammation state; there is a risk of concurrent SCVS. At the same time, in order to further explore and visualize the predictive effectiveness of SIRI, in this study, a nomogram predictive model of SCVS was built based on the level of SIRI inflammation and other related risk factors. It has been verified that the C-index and the area under the ROC curve of the model are all good; it has reliable predictive efficiency and consistency and is suitable for clinical use. For example, a patient has a history of hypertension, Hunt-Hess grade IV-V at the time of admission, modified Fisher grade IV-V, combined with ventricular hemorrhage, *TG* = 1.46*mmol*/*L*, and *SIRI* = 4.85 × 10^9^/*L*, through the nomogram model scoring line; the patient's total score is 365 points (94 + 73 + 98 + 87 + 0 + 39); the corresponding risk prediction value is 0.754; that is, the patient has a 75.4% probability of complicated SCVS. Nomogram can quickly and intuitively predict the probability of patients with SCVS and achieve individualized prediction [20].

## 4. Conclusion

Retrospectively analyze the data of aSAH patients admitted to a hospital, discuss the value of SIRI's assessment of SCVS, and based on the SIRI level to build a simple and reliable nomogram prediction model, nomogram can quickly and intuitively predict the occurrence probability of patients with SCVS and realize individualized prediction. SIRI is closely related to SCVS after aSAH, and the nomogram model constructed with SIRI will optimize the prediction efficiency and improve the ability of early identification and screening of SCVS.

## Figures and Tables

**Figure 1:** The ROC curve of SIRI predicting the occurrence of SCVS in aSAH patients after surgery.

**Table 1:** Comparison of general data of patients in SCVS group and non-SCVS group.

Factor		SCVS group	Non-SCVS group	*t*/*x*^2^/*z*	*P*
Age		58.31 ± 13.415	55.37 ± 11.88	-0.976	0.331

Gender	Man	5 (26.31)	40 (37.75)	0.913	0.341
	Women	14 (73.69)	66 (62.24)		

Smoking	Yes	10 (52.62)	24 (22.63)	7.318	0.007
	No	9 (47.38)	82 (77.35)		

Drinking	Yes	7 (36.82)	24 (22.65)	1.742	0.187
	No	12 (63.14)	82 (77.38)		

Hypertension	Yes	15 (78.94)	36 (33.97)	13.499	0.001
	No	4 (21.051)	70 (66.07)		

**Table 2:** Comparison of various indicators between CVS group and non-SCVS group.

Factor		SCVS group	Non-SCVS group	*t*/*x*^2^/*z*	*P*
Hunt-Hess classification	IV-V	11 (57.88)	28 (26.41)	7.439	0.007
	I-III	8 (42.12)	78 (73.57)		

Number of aneurysms	Multiple shots	5 (26.33)	12 (11.31)	3.082	0.078
	Single shot	14 (73.69)	94 (88.69)		

Merged IVH	Yes	11 (57.88)	23 (21.71)	10.662	0.001
	No	8 (42.10)	83 (78.32)		

Improved fisher classification	IV-V	12 (63.15)	25 (23.59)	12.109	0.001
	I-III	7 (36.86)	81 (76.43)		

TG		1.81 (1.39, 2.08)	1.28 (0.93, 1.64)	-3.414	0.001
Monocyte count		0.61 (0.51, 0.72)	0.41 (0.28, 0.63)	-3.231	0.001
SIRI		3.91 (1.94, 6.93)	2.39 (1.53, 4.54)	-2.282	0.021

**Table 3:** Multivariate analysis of SCVS in postoperative patients with aSAH.

Factor	*β*	Standard error	Woldx^2^	OR value	95% CI	*P* value
Hypertension	2.298	0.853	7.172	4.653	1.847-23.584	0.006
Hunt-Hess classification	1.553	0.771	4.100	3.778	1.052-16.716	0.042
Merged IVH	2.305	0.956	5.807	4.035	1.538-20.453	0.017
Improved Fisher classification	2.566	0.967	7.055	5.021	1.959-28.554	0.009
TG	1.611	0.568	8.017	3.001	1.641-10.249	0.005
SIRI	0.332	0.163	4.075	1392	1.011-1.932	0.043

## Data Availability

The data used to support the findings of this study are available from the corresponding author upon request.
